This article has been retracted.

# *In Silico* Characterization of Growth Differentiation Factors as Inhibitors of TNF-Alpha and IL-6 in Immune-Mediated Inflammatory Disease Rheumatoid Arthritis

**DOI:** 10.1155/2021/5538535

**Published:** 2021-03-26

**Authors:** Ghulam Mustafa, Hafiza Salaha Mahrosh, Rawaba Arif

**Affiliations:** Department of Biochemistry, Government College University, Faisalabad 38000, Pakistan

## Abstract

Tumor necrosis factor alpha (TNF-*α*) plays a critical role in the progression of inflammation and affects the cells of the synovial membrane. Another key factor in the progression of rheumatoid inflammation is interleukin-6 (IL-6). Both TNF-*α* and IL-6 promote the proliferation of synovial membrane cells thus stimulating the production of matrix metalloproteinases and other cytotoxins and leading towards bone erosion and destruction of the cartilage. Growth differentiation factor-11 (GDF11) and growth differentiation factor-8 (GDF8) which is also known as myostatin are members of the transforming growth factor-*β* family and could be used as antagonists to inflammatory responses which are associated with rheumatoid arthritis. In the current study, to elucidate the evolutionary relationships of GDF11 with its homologs from other closely related organisms, a comprehensive phylogenetic analysis was performed. From the phylogram, it was revealed that the clade of Primates that belong to superorder Euarchontoglires showed close evolutionary relationships with order Cetartiodactyla of the Laurasiatheria superorder. Fifty tetrapeptides were devised from conserved regions of GDF11 which served as ligands in protein-ligand docking against TNF-*α* and IL-6 followed by drug scanning and ADMET profiling of best selected ligands. The peptides SAGP showed strong interactions with IL-6, and peptides AFDP and AGPC showed strong interactions with TNF-*α*, and all three peptides fulfilled all the pharmacokinetic parameters which are important for bioavailability. The potential of GDF8 as an antagonist to TNF-*α* and IL-6 was also explored using a protein-protein docking approach. The binding patterns of GDF8 with TNF-*α* and IL-6 showed that GDF8 could be used as a potential inhibitor of TNF-*α* and IL-6 to treat rheumatoid arthritis.

## 1. Introduction

The immune system is a collection of chemicals, cells, and pathways that protect the cells from foreign invaders. Beyond chemical and physical barriers to pathogens, the immune system has two fundamental pillars in line of defense which include innate immunity and adaptive immunity [1]. Innate immunity is a nonspecific rapid immune response activated within minutes to hours with the lack of immunologic memory. On the other hand, adaptive immunity is an antigen-dependent response activated upon the subsequent exposure of host cells to antigens. There is synergy between the events in innate immunity and adaptive immunity, and any defect in either system provokes severe problems and diseases such as autoimmune diseases, inflammations, and immunodeficiency disorders [2].

The immune system preserves homeostasis in immune integrity to protect the host cells from infectious agents. Furthermore, the immune system undergoes processed pathways to initiate self-tolerance to avoid the destruction of tissues or cells of the host immune system. The impairment of the self-tolerance mechanism leads towards the onset of severe autoimmune disorders [3]. Mounting evidence has clearly demonstrated the relation of innate immunity responses in initiation, progression, and maintenance of different autoimmune disorders including lupus erythematosus, rheumatoid arthritis, Alzheimer's disease, Addison's disease, and type I diabetes mellitus [2]. Autoimmunity involves the self-destruction of own tissues by the production of abnormal responses due to self-reactive T-cells, cytokines, and autoantibodies. To design potential drugs and targets, these self-reactive species are the main focus to maintain different autoimmune disorders [4].

In this study, our main focus was on the systemic autoimmune disease rheumatoid arthritis (RA). Rheumatoid arthritis (RA) is an autoimmune disease characterized by synovial inflammation, decalcification, bone erosion, and destruction of cartilage which result in joint impairment. Currently, there are five main classes of drugs that have been in practice in RA therapy including analgesics, glucocorticoids, biologic disease-modifying antirheumatic drugs (bDMARDs), nonbiologic disease-modifying antirheumatic drugs, and nonsteroidal anti-inflammatory drugs (NSAIDs). The most common biological disease-modifying antirheumatic drugs are TNF-*α* inhibitors. Despite many drug therapies, the RA patients did not get any significant clinical benefits from these agents [5].

On the basis of sequence identity, shared inhibitors, and receptor utilization, the members of the transforming growth factor-*β* (TGF-*β*) family may be divided into three subclasses, i.e., TGF-*β*, bone morphogenetic protein (BMP)/GDF, and activin/inhibin [6, 7]. A similar protein fold has been observed in all proteins of the TGF-*β* family, and efforts have been made to understand the structural basis of these individual ligands for their differential signaling. Growth differentiation factor-11 (GDF11) also known as bone morphogenetic protein 11 (BMP11) is a member of the transforming growth factor-*β* (TGF-*β*) family [8]. From this family, GDF11 and GDF8 (also known as myostatin) have been found to be the most closely related members and emerged through a gene duplication event in an ancestral gene after the point when divergence of amphioxus occurred from vertebrates [9]. It has been observed that both GDF8 and GDF11 bind with type II receptors of activin which trigger signaling via the Smad2/3 pathway after subsequent phosphorylation of these receptors [10].

The aim of this study includes the investigation of potential tumor necrosis factor alpha (TNF-*α*) and interleukin-6 (IL-6) inhibitors which could be used in RA maintenance. Currently, the attenuation of inflammatory responses has attracted the attention of researchers in the field of many inflammatory disorders. Recently, the therapeutic effects of GDF11 in mouse models as an antagonist of inflammatory responses associated with RA have been explored [11]. In the current study, we therefore explored the inhibitory nature of GDF11 against the proinflammatory cytokines responsible for rheumatoid arthritis.

## 2. Materials and Methods

### 2.1. Phylogenetic Analysis

Human *GDF11* gene sequence was retrieved from the NCBI nucleotide database and analyzed using BLAST (Basic Local Alignment Search Tool) [12] available on the NCBI website (http://www.ncbi.nlm.nih.gov/). Along with *GDF11* gene sequence of *Homo sapiens*, seventy-four most similar reported sequences of *GDF11* from different mammals were also retrieved from GenBank for phylogenetic systematics. All sequences were aligned using ClustalX and imported into the MEGA7 program [13] for manual alignment. A Neighbor-Joining (NJ) phylogenetic tree was reconstructed using MEGA7 with 100 bootstrap replicates.

### 2.2. Ligand-Based Molecular Docking

A ready-to-dock library of 50 ligands was prepared and docked against tumor necrosis factor alpha (TNF-*α*) and interleukin-6 (IL-6) with the help of Molecular Operating Environment (MOE) software.

### 2.3. Ligand Selection and Database Preparation

The protein sequence of GDF11 was retrieved from NCBI's Entrez Protein under accession No. O95390.1. MEME Suite was used to predict three motifs from nine selected homologs of GDF11 [14, 15]. The chemical structures of 50 tetrapeptides were drawn from the consensus sequences of predicted motifs using ACD ChemSketch and saved in MOL format. All the tetrapeptides were minimized and saved into the MOE database in .mdb format for docking studies.

### 2.4. Retrieval and Optimization of Receptor Proteins

Three-dimensional structures of TNF-*α* (PDB ID: 6OP0) and IL-6 (PDB ID: 5FUC) were retrieved from Protein Data Bank (PDB) and optimized by removing water molecule, addition of hydrogen atoms, energy minimization, and 3D protonation using MOE software. The ready-to-dock database of 50 tetrapeptides was docked counter to TNF-*α* and IL-6 separately. The top five interaction conformations of each receptor protein were selected on the basis of binding patterns and energy conformations.

### 2.5. Protein-Ligand Docking

Active sites of receptor proteins were predicted by a site finder tool of MOE with default parameters. The prepared database of 50 tetrapeptides from the conserved sequences of GDF11 was docked counter to receptor proteins separately using MOE. The docking program of MOE provides the top conformations on the basis of maximum occupancy of binding pocket and minimum energy structure. The top five ligands from each protein-ligand docking study were selected on the basis of *S*-scores and kept aside for further verification through drug scan analysis.

### 2.6. Drug Scanning and ADMET Profiling

Lipinski's rule of five explores the therapeutic nature of selected drug molecules by distinguishing the drug-like and nondrug-like properties of drug candidates. The durability of hit compounds was evaluated using the online server SwissADME [16]. The ADMET (metabolism, distribution, excretion, absorption, and toxicity) attributes of target molecules were discovered using admetSAR server [17]. Only those ligands were considered to be the potential or lead drug candidates that accomplished all the ADMET models successfully.

### 2.7. Protein-Protein Docking

Appropriate interactions between the member of TGF-*β* and TNF-*α* and IL-6 are necessary to check binding residues between them and to inhibit the residues of receptor protein(s). In this study, the chain A of myostatin (PDB ID: 6UMX) was selected as a template and downloaded from PDB to dock against receptor proteins TNF-*α* (PDB ID: 6OP0) and IL-6 (PDB ID: 5FUC). The inhibitors of TNF-*α* and IL-6 have been extensively studied and researched due to their role in reduction of inflammatory response in autoimmune disorders. The HADDOCK server was used to dock myostatin with TNF-*α* and IL-6 [18]. To visualize the interactions, the educational version of PYMOL was used [19]. Moreover, the online database PUBsum was used to demonstrate the interacting residues involved in protein-protein interactions [20].

## 3. Results and Discussion

Basic Local Alignment Search Tool (BLAST) is still the most popular search algorithm and can accommodate nucleotide or protein sequences. BLAST was used to identify local regions of similarity and statistical significance of *GDF11* nucleotide sequences from selected organisms. Multiple sequence alignment was also performed through Geneious [21] (Fig S1 of Supplementary file). The truncated sequences were deleted, and longer sequences were shortened in the multiple sequence alignment to make them all equal in length.

### 3.1. Analysis of *GDF11* Phylogenetic Tree

To establish the evolutionary relationships, a phylogenetic tree of the *GDF11* gene from seventy-six members of the Eutheria clade of mammals with maximum identity including *H. sapiens* was reconstructed (Figure 1). The evolutionary history was inferred using the Neighbor-Joining method [22, 23]. The percentage of replicate trees in which the associated taxa clustered together in the bootstrap test (100 replicates) is shown next to the branches [24, 25]. The tree was drawn to scale, with branch lengths in the same units as those of the evolutionary distances used to infer the phylogenetic tree. The evolutionary distances were computed using the Kimura 2-parameter method [26] and are in the units of the number of base substitutions per site. Overall mean distance was found to be 0.052. The tree is fully in accordance with the classification system, and all organisms appeared in their respective clades and subclades. The organisms divided themselves under three superorders, i.e., Euarchontoglires, Laurasiatheria, and Afrotheria, with two, four, and five orders covered, respectively. *Oryctolagus cuniculus* has appeared in Glires and *Homo sapiens* in Primates orders under the same superorder of Euarchontoglires. From the phylogeny of *GDF11*, it was inferred that *O. cuniculus* had the strongest evolutionary relationship with *Ochotona princeps* while *H. sapiens* with *Gorilla gorilla gorilla*. Some interesting observations were also found in the phylogeny of *GDF11*. The Primates order that belongs to superorder Euarchontoglires is showing more identity with order Cetartiodactyla of the Laurasiatheria superorder, inferring that there would be some evolutionary closeness between two orders. The organisms of order Chiroptera have not appeared in a single clade and are divided into two small clades, i.e., Chiroptera I and Chiroptera II. Chiroptera II is showing more closeness with the Perissodactyla order hypothesizing that the organisms under both clades have strong evolutionary relationships.

A detailed phylogenetic analysis for GDF11 sequences was not found previously, and therefore, in this study, we conducted a comprehensive phylogenetic analysis. In our phylogenetic analysis, the mammalian GDF11 clades were divided into different clades on the basis of their suborders. Biga et al. [27] also conducted a phylogeny of GDF11 using protein sequences. They found that GDF11 from mammals clustered with that of zebrafish and also found that all myostatin and GDF11 sequences were grouped together showing high identity between both proteins. In another study [28], GDF11 and myostatin in vertebrates were found to be more closely related to each other than piscine myostatin when a phylogenetic analysis of GDF11 and myostatin was performed.

More than 30 ligands have been reported from the TGF-*β* family, which are structurally related but functionally distinct. The family has 3 subclasses, i.e., TGF-*β*s, BMPs, and activin/myostatins. From the TGF-*β* family, GDF11 and GDF8 (myostatin) have 90% sequence identity within their mature signaling domain and both are members of the activin/myostatin subclass [29]. Talking about the function of GDF11, it is essential for the development of mammals and has been recognized for the regulation of aging of various tissues. GDF8, however, has been found as a strong negative regulator of muscle growth and modulates various metabolic processes [30].

Other differences in GDF11 and GDF8 are also studied and observed that GDF11 mRNA is found largely in various tissues [31] but most abundant in the kidney and spleen [32], whereas GDF8 mRNA is mainly found in cardiac and skeletal muscles. Both proteins are found in the bloodstream, and the functional effects of their circulation are still not clear, but it has been suggested that their presence may act as hormonal signals. It was suggested that a number of features and functions of both GDFs could overlap because of their high sequence similarity, but the latest studies have shown that both ligands have different functions [29]. Due to identical residues in the region, both proteins possibly bind type II receptors in the same fashion, but the residues have been found divergent in the prehelix loop and wrist helix between GDF11 and GDF8 conferring that the binding of type I receptors might be different in both ligands [33].

Because of high sequence similarity and conservation between GDF11 and GDF8, the functions of both the ligands were assumed to be similar [34]. It is likely that much of this assumption reflects the fact that GDF11 is a comparatively understudied ligand of the TGF-*β* family as compared to other members especially GDF8, and thus, the tools to study the biology of GDF11 are continuously evolving. Therefore, we have studied GDF11 in more detail and gave its comprehensive evolutionary relationships through its phylogeny.

### 3.2. Devising of Tetrapeptides as Ligands

Protein BLAST (BLASTp) was used to explore homologs of GDF11 based on query converge. MEME Suite was then used to explore three motifs from the selected homologs. The most conserved 50 tetrapeptides were devised from the selected motifs as ligand molecules and saved in the MOE database.

### 3.3. Protein-Ligand Docking

Molecular docking is a computer-aided drug discovery used to predict the perfect orientation of ligand molecules. This study includes a ready-to-dock library of 50 tetrapeptides devised from GDF11 and docked against tumor necrosis factor alpha and interleukin-6. The top hit compounds were selected on the bases of *S*-scores and energy validations for further analyses.

### 3.4. Interaction Analyses

According to given commands, MOE gave different confirmations of all ligands. The top five ligands from each protein-ligand study were selected as hit compounds on the basis of *S*-scores and binding residues. For TNF-*α*, the peptide TETV exhibited the best *S*-score (i.e., -14.7233) and showed interactions with amino acids Ser147 and His15 of the binding pocket (Figure 2). Other peptides (i.e., ISMA, ANPR, AFDP, and AGPC with *S*-scores -14.4874, -14.4748, -14.1934, and -13.6792, respectively) also showed interactions with active amino acids of the binding site (Figs 2S to 5S, respectively, of Supplementary file).  Table 1 is showing peptides with their docking scores and interacting residues of TNF-*α*.

Other receptor protein interleukin-6 is a pleiotropic anti-inflammatory myokine and proinflammatory cytokine encoded by the IL-6 gene in humans. In our study, the peptide AQET exhibited the best *S*-score (-11.4547) with interactive amino acid residues (i.e., Met67 and Glu172) of the binding pocket (Figure 3). Four peptides (i.e., DGSP, TETV, SAGP, and GSAG with *S*-scores of -10.9771, -10.2757, -10.0603, and -9.9370, respectively) showed excellent binding interactions with active amino acids (Figs 6S to 9S, respectively, of Supplementary file).  Table 1 is showing peptides with their docking scores and interacting residues of IL-6.

The elevated level of plasma IL-6 is associated with insulin resistance in diabetes mellitus [35]. IL-6 binds to the receptor on the cellular surface and forms an IL-6/sIL-6R complex that leads towards activation of cells. IL-6 also promotes T-cell differentiation and at the same time collaborates with TNF-*α* and IL-1 to induce systemic inflammatory response [36]. TNF-*α* is also a proinflammatory cytokine used by the immune system in a defense mechanism to induce inflammation against pathogenic response. The deregulation or elevated signaling of TNF-*α* alters the balance of T-cells thus leading towards the inflammatory diseases such as inflammatory bowel disease, rheumatoid arthritis (RA), and ankylosing spondylitis (AS). Collectively with TNF-*α*, the role of IL-6 has been studied in humans and different animal models to understand the phenomena of autoimmunity [37]. Thus, there is a dire need for new drugs to regulate the cytokine signaling and reduce the inflammatory responses to treat autoimmune disorders.

### 3.5. Drug Scan and ADMET Screening

The Lipinski rule of five distinguishes the drug-like and nondrug-like molecules based on five parameters (i.e., molecular mass: ≤500 daltons, hydrogen bond donor: <5, hydrogen bond acceptor: <10, molar refractive index: 40-130, and partition coefficient (log *P*): ≤5). The three peptides SAGP, AFDP, and AGPC showed no deviation and fully accomplished the criteria of potent drug candidates. The remaining peptides AQET, DGSP, TETV, SAGP, GSAG, ISMA, and ANPR showed only one violation of Lipinski's rule of five (Table 2). The ADMET-based drug profiling is necessary to estimate the bioavailability of drug candidates. The ADMET study evaluates the hit compounds using different threshold values to estimate the absorption of leading compounds. In the current study, all the selected compounds were found to be noncarcinogens and non-Ames toxic (Table 3). Based on overall drug profiling, these ligands could be used as potential inhibitors of TNF-*α* and IL-6.

### 3.6. Protein-Protein Docking

Protein-protein docking is the prediction of binding complexes between two proteins to demonstrate the protein-protein interference. The HADDOCK server was used to perform template-based docking and to predict the interacting residues through hybrid algorithms. In this study, the docking analysis was performed to dock myostatin (GDF8) protein (which showed >85% sequence identity with GDF11) with TNF-*α* and IL-6. The results revealed good binding patterns and interactions between amino acids of two protein complexes. The HADDOCK binding score of GDF-TNF-*α* was found to be -62.2 kcal/mol and that of GDF-IL-6 was found to be -48.1 kcal/mol. The interactions between GDF8 and TNF-*α* are shown in Figure 4 while interactions between GDF8 and IL-6 are shown in Figure 5.

The hydrogen bonds between GDF8 and both target proteins are shown in red stick representation. In the case of GDF-TNF-*α* interactions, it was observed that the active amino acids of GDF8 were involved in six hydrogen bonds with TNF-*α*; meanwhile, 16 hydrogen bonds were observed in GDF-IL-6 interactions. The online database PUBsum also demonstrates the hydrogen bonding along with disulfide bonds between the active amino acids of these protein complexes. The overall results and binding patterns of GDF8 with TNF-*α* and IL-6 indicated that GDF8 could be used as a potential inhibitor of TNF-*α* and IL-6 receptor proteins.

The molecular docking approach predicts the best orientation of ligands binding with particular amino acids of the binding pocket of receptor molecules [15]. Molecular docking is the major section of drug discovery as it predicts the biological interactions and bioavailability of hit compounds. Computational drug discovery is the most economic and effective route of *in silico* drug designing [38]. Based on the type of ligands, docking can be classified into many types like protein-small molecule (ligand) docking, protein-protein docking, and protein-nucleic acid docking [39]. In the current study, we used two approaches (i.e., ligand-based protein docking and protein-protein docking) of TGF-*β* members counter to two target proteins such as tumor necrosis factor alpha and interleukin-6.

Human TNF-*α* is 17 kDa in size, nonglycosylated, and encoded by genes on 6p23-6q12. TNF-*α* mainly involves in a variety of functions including phagocytosis of neutrophilic granulocytes, cytolysis and cytostasis of many tumor cells, and modulations of many other proteins such as IL-1 and IL-6 [40]. TNF-*α* is a pleiotropic cytokine, a key mediator of chronic and acute inflammations secreted by macrophages, neutrophils, and T-cells [41]. With the combination of IL-6 and IL-1, TNF-*α* performs a variety of functions including endothelium alterations, inhibition of anticoagulatory mechanisms, and B-cell differentiation and proliferation. Although TNF-*α* is a necessary cytokine, its overexpression or deregulation is associated with different autoimmune diseases [40].

Interleukin-6 is a proinflammatory cytokine and an anti-inflammatory myokine transiently produced by the host immune system as the result of an infection. Human IL-6 protein is of ∼20 kDa and contains 212 amino acids encoded by genes on chromosome 7p21 [42]. Interleukin-6 plays a critical role in host immunity, acute-phase reactions, and hematopoiesis. Although the expression and regulation of IL-6 have been completely controlled by posttranscriptional mechanisms, any mutation in the IL-6 regulatory mechanism leads towards chronic inflammation and autoimmunity [43]. Under the presumption that IL-6 and TNF-*α* cause autoimmunity, therefore, several drugs have been designed to treat autoimmune diseases. All the anti-TNF-*α* and IL-6 therapies have been totally designed to negate the TNF-*α* and IL-6 activity by blocking the TNF transcription and NF-mediated downstream signaling [40, 44].

The blockage of TNF-*α* and IL-6 has been expected as an effective strategy for the treatment of many autoimmune disorders. Many IL-6 antibodies have been developed to inhibit the IL-6 signaling and transduction pathways. Among all the designed antibodies, anti-IL-6RAb commonly known as tocilizumab showed efficient results in clinical trials for rheumatoid arthritis as anti-IL-6RAb. The tolerability profiles of anti-IL-6RAb monotherapy proved safe and potent and therefore could be used as an anti-RA antibody. Several clinical studies supported the inhibitory nature of tocilizumab as an anti-IL-6 receptor monoclonal antibody and showed astonishing efficacy in RA [42, 45]. In another study, suppression of proinflammatory cytokine responses by targeting the JAK/STAT pathway has been demonstrated as a therapeutic option in saphenous vein graft failure. The results of different clinical trials including suppression of cytokine signaling (SOCS3) showed that it appears as a major contributor to suppression of unwanted vascular inflammation and proliferation [46].

Wang et al. [47] demonstrated the dual nature of different ligands as potential inhibitors of TNF-*α* and IL-6. The results of their study showed that two molecules (i.e., ZINC19701771 and ZINC06576501) exhibited the best binding pattern and pharmacological properties and therefore could be served as potential candidates for the development of an anti-RA drug. In the current study, we used two approaches of molecular docking to check the therapeutic nature of two members of the TGF-*β* family (i.e., GDF11 and GDF8/myostatin) as antagonists of TNF-*α* and IL-6. In the first approach, ligand-based docking was performed and 50 tetrapeptides were devised from conserved regions of GDF11 counter to two inflammatory receptor proteins such as TNF-*α* and IL-6. On the basis of confirmations and orientation of ligands, the top five peptide molecules were selected for further pharmacokinetic analysis. The peptide TETV with the best *S*-score (-14.7233) showed interactions with amino acids Ser147 and His15 present in the binding pocket of TNF-*α*. Similarly, the peptide AQET was found with the top *S*-score (-11.4547) and interacted with amino acids Met67 and Glu172 of the binding pocket of IL-6 receptor protein.

The drugability test of all selected peptides fulfilled the criteria of being potential drug candidates by following the Lipinski rule of five. Out of ten selected peptides, three peptides (i.e., SAGP, AFDP, and AGPC) followed all the five parameters of Lipinski's rule of five while other peptides showed only one violation. The ADMET profiling of all leading compounds was also found satisfactory as all hit compounds were revealed to be noncarcinogens and non-Ames toxic. Therefore, based on overall drug profiling, these ligands could be used as potential inhibitors of TNF-*α* and IL-6.

In the next approach, we used protein-protein docking via the HADDOCK server to check the binding interactions of GDF8 with TNF-*α* and IL-6. The binding score of GDF-TNF-*α* was found to be -62.2 kcal/mol with 6 hydrogen bonds between active residues, and GDF-IL-6 showed a binding score of -48.1 kcal/mol with 16 hydrogen bonds. Later, all these interactions were confirmed by comparing the results of HADDOCK with those of PUBsum. From results of this study, it can be concluded that both members of TGF-*β* can be used as therapeutic agents against two main inflammatory cytokines (i.e., TNF-*α* and IL-6) for the treatment of rheumatoid arthritis. This study can be used as a reference to explore more aspects and involvement of GDF8 and GDF11 in the treatment of autoimmune disorders.

## 4. Conclusion

From a comprehensive phylogenetic analysis of GDF11, protein-ligand and protein-protein docking, the potential of TGF-*β* members (GDF11 and GDF8) as drug inhibitors of TNF-*α* and IL-6 receptor proteins has been revealed. Three tetrapeptides (i.e., SAGP: against IL-6; AFDP and AGPC: against TNF-*α*) devised from GDF11 with good docking scores fulfilled all the criteria of being good drug candidates. TNF-*α* and IL-6 are the proinflammatory cytokines that regulate the inflammatory responses and signaling upon infections. In the case of deregulation of these cytokines, the circumstances lead towards the onset of autoimmunity and resistance in self-tolerance. In the current study, different approaches were employed to explore the inhibitory nature of GDF11 and GDF8 counter to TNF-*α* and IL-6. The energy validations and scoring of molecular docking results showed the potential of GDF11 and GDF8 as drug candidates with no toxicity.

## Figures and Tables

**Figure 1:** Phylogenetic relationships of the *GDF11* gene in selected organisms. The tree is labeled on the basis of orders and suborders of selected animals. The animals of the same suborder cladded together.

**Figure 2:** Interactions (a) and binding patterns (b) of TETV with TNF-*α*.

**Figure 3:** Interactions (a) and binding patterns (b) of AQET with IL-6.

**Figure 4:** Protein-protein interactions between myostatin and TNF-*α*. (a) GDF8/TNF-*α* docked complex in cartoon representation is shown at the top. Myostatin is shown in green while TNF-*α* is shown in blue. Interacting residues of the GDF8/TNF-*α* complex are shown in red color stick representation. (b) All interacting residues of GDF8 and TNF-*α*. Blue color: H-bonds, red color: salt bridges, yellow color: disulfide bonds, orange color: other contacts. Hydrogen bonds are shown with blue lines. The colors of interacting residues are representing properties of amino acids (i.e., blue: positive, red: negative, green: aliphatic, grey: aliphatic, pink: aromatic, orange: Pro/Gly, and yellow: Cyc).

**Figure 5:** Protein-protein interactions between myostatin and IL-6. (a) GDF8/IL-6 docked complex in cartoon representation is shown at the top. Myostatin is shown in green, and IL-6 is shown in yellow. Interacting residues of the GDF8/IL-6 complex are shown in red color stick representation. (b) All interacting residues of GDF8 and IL-6. Blue color: H-bonds, red color: salt bridges, yellow color: disulfide bonds, and orange color: nonbonded contacts. Hydrogen bonds are shown with blue lines. The colors of interacting residues are representing properties of amino acids (i.e., blue: positive, red: negative, green: aliphatic, grey: aliphatic, pink: aromatic, orange: Pro/Gly, and yellow: Cyc).

**Table 1:** Top interactions of GDF11 tetrapeptides with TNF-*α* and IL-6 as receptor proteins.

Sr. No.	Peptide	Receptor	*S*-score	Interacting residues
1	TETV	TNF-*α*	-14.7233	Ser147, His15
2	ISMA		-14.4874	Gly148
3	ANPR		-14.4748	Arg32, Glu146, Val150
4	AFDP		-14.1934	Ala33, Ser147
5	AGPC		-13.6792	His15, Gln149, Val150, Ser147
6	AQET	IL-6	-11.4547	Met67, Glu172
7	DGSP		-10.9771	Met67, Arg179
8	TETV		-10.2757	Glu172, Arg179, Arg168
9	SAGP		-10.0603	Glu172, Arg179, Ser169, Ser176
10	GSAG		-9.9370	Glu172, Glu172, Arg179

**Table 2:** Pharmacokinetic parameters important for bioavailability of compounds drug-likeness properties of selected peptides.

Sr. No.	Peptides	Receptor	Molecular properties^†^					
			Mass (<500 D)	HBD (≤5)	HBA (≤10)	Log *P* (<5)	Molar refractivity (40-130)	Violations
1	SAGP	IL-6	330.34	5	7	-2.32	81.15	0
2	AFDP	TNF-*α*	448.47	5	8	-0.75	115.86	0
3	AGPC	TNF-*α*	346.40	4	6	-1.58	87.91	0
4	TETV	TNF-*α*	448.47	10	8	-2.25	106.22	1
5	AQET	IL-6	447.44	8	10	-2.93	103.16	1
6	GSAG	IL-6	290.27	6	7	-2.92	64.83	1
7	ISMA	TNF-*α*	420.52	6	7	-0.93	106.07	1
8	ANPR	TNF-*α*	456.50	8	8	-3.21	116.03	1
9	DGSP	IL-6	374.35	6	9	-2.95	87.73	1

HBD: hydrogen bond donors; HBA: hydrogen bond acceptors; log *P*: the logarithm of octanol/water partition coefficient.

**Table 3:** ADMET profiling of the best selected peptides.

	Peptides								
	AQET	DGSP	TETV	SAGP	GSAG	ISMA	ANPR	AFDP	AGPC
Absorption									
BBB	+	+	+	+	+	+	+	−	+
HIA	−	−	−	−	−	−	−	−	−
Caco-2 permeability	−	−	−	−	−	−	−	−	−
PGS	NS	Substrate	NS	NS	NS	Substrate	Substrate	Substrate	Substrate
PGI	NI	NI	NI	NI	NI	NI	NI	NI	NI
ROCT	NI	NI	NI	NI	NI	NI	NI	NI	NI
Metabolism									
CYP3A4 substrate	NS	Substrate	NS	Substrate	NS	NS	Substrate	Substrate	Substrate
CYP2C9 substrate	NS	NS	NS	NS	NS	Substrate	NS	NS	NS
CYP2D6 substrate	NS	NS	NS	NS	NS	NS	NS	NS	NS
CYP3A4 inhibition	NI	NS	NI	NS	NI	NI	NI	NI	NI
CYP2C9 inhibition	NI	NI	NI	NI	NI	NI	NI	NI	NI
CYP2C19 inhibition	NI	NI	NI	NI	NI	NI	NI	NI	NI
CYP2D6 inhibition	NI	NI	NI	NI	NI	NI	NI	NI	NI
CYP1A2 inhibition	NI	NI	NI	NI	NI	NI	NI	NI	NI
Toxicity									
AMES toxicity	NAT	NAT	NAT	NAT	NAT	NAT	NAT	NAT	NAT
Carcinogens	NC	NC	NC	NC	NC	NC	NC	NC	NC

BBB: blood-brain barrier; HIA: human intestinal absorption; PGS: P-glycoprotein substrate; PGI: P-glycoprotein inhibitor; ROCT: renal organic cation transporter; NS: nonsubstrate; NI: noninhibitor; NAT: non-Ames toxic; NC: noncarcinogenic.

## Data Availability

The data used to support the findings of this study are available from the corresponding author upon request.

## Supplementary Materials

Supplementary Materials Fig S1: multiple sequence alignment of GDF11 gene from selected organisms to show sequence similarities/differences. Fig 2S: interactions (a) and binding patterns (b) of ISMA with TNF-*α*. Fig 3S: interactions (a) and binding patterns (b) of ANPR with TNF-*α*. Fig 4S: interactions (a) and binding patterns (b) of AFDP with TNF-*α*. Fig 5S: interactions (a) and binding patterns (b) of AGPC with TNF-*α*. Fig 6S: interactions (a) and binding patterns (b) of DGSP with IL-6. Fig 7S: interactions (a) and binding patterns (b) of TETV with IL-6. Fig 8S: interactions (a) and binding patterns (b) of SAGP with IL-6. Fig 9S: interactions (a) and binding patterns (b) of GSAG with IL-6.
